# Dynamic risk spillover effect and path of risk transmission across industrial sectors in China during COVID-19 epidemic

**DOI:** 10.1371/journal.pone.0292859

**Published:** 2023-10-13

**Authors:** Lin Ling, Hayat Khan, Jiang Lingwei, Li Qiumei, Zhang Zuominyang, Itbar Khan

**Affiliations:** 1 School of Business Administration, Guangxi University of Finance and Economics, Nanning, China; 2 School of Economics and management, Zhejiang University of Science and Technology, Hangzhou, China; 3 Graduate School, Guangxi University of Finance and Economics, Nanning, China; 4 College of Economics, Shenzhen University, Shenzhen, China; University of Galway, Ireland / Anhui University of Finance and Economics, CHINA

## Abstract

Understanding the dynamic link between the development of COVID-19 pandemic and industry sector risk spillovers is crucial to explore the underlying mechanisms by which major public health events affect economic systems. This paper applies ElasticNet method proposed by Diebold and Yilmaz (2009, 2012, 2014) to estimate the dynamic risk spillover indicators of 20 industrial sectors in China from 2016 to 2022, and systematically examines the impact of industry risk network fluctuations and the transmission path caused by COVID-19 shock. The findings reveal that risk spillovers of Chinese industries show a dynamic change of "decline-fluctuation-rebound" with the three phases of COVID-19 epidemic. At the beginning of the epidemic, machinery and equipment, paper and printing, tourism and hotels, media and information services, and agriculture were the exporters of epidemic risk, while materials, transportation equipment, commercial trade, health care, and environmental protection were the importers of epidemic risk; However, as the epidemic developed further, the direction and effect of risk transmission in the industry was reversed. Examining the network characteristics of the pair sectors, we found that under the epidemic shock, the positive risk spillover from tourism and hotels, culture, education and sports to consumer goods, finance, and energy industries was significantly increased, and finance and real estate industries were affected by the risk impact of more industries, while the number of industries affected by information technology and computer industry was significantly reduced. This paper shows that there is inter-industry risk transmission of the COVID-19 epidemic shock, and the risk transmission feeds back in a cycle between industries as the epidemic develops, driving the economy into a vicious circle. The role of the service sector in blocking the spread of negative shocks from the epidemic should be emphasized and brought into play to avoid increasing the overall economic vulnerability. This study will help to deepen the understanding of scholars and policy makers on the network transmission effects of the epidemic.

## 1. Introduction

The development of COVID-19, which suddenly bust out in 2020, has been developing for three years. Although China has adjusted the COVID-19 infection to Category B, and social face-to-face epidemic control measures tend to relax, the situation of the epidemic situation may still occur in the future. Large-scale infectious disease outbreaks have always been public health emergencies that seriously threaten human health and social security [1–4], and have a serious impact on the economic operation system [5, 6]. The deep understanding of the dynamic link between the development of COVID-19 pandemic and industry sector risk spillovers is crucial to explore the underlying mechanisms by which major public health events affect economic systems. Early studies focused on retrospective analysis of major infectious disease events in history and examined the overall impact of major infectious diseases on economic and social development. For example, Hirshleifer [7] delved into the outbreak of the Black Death in Western Europe in 1348 and its short and long-term macroeconomic impacts, pointing out that sudden disasters caused a certain degree of social disruption in the short term and slowed down the economic growth of Western Europe in the following century in the long run. Alfani and Percoco [8] used data on plague mortality in 56 cities from 1575–1700, systematically examined the long-term economic impact of the plague on Italian from 1629–1630, and found that the plague caused long-term damage to the size of Italian urban population and urbanization rates, triggered a decline in the Italian economy. Research on the impact of major infectious disease events on economic development in China began in 2003 after the outbreak of SARS in China. Lee and McKibbin [9] estimated the economic impact of the severe acute respiratory syndrome (SARS) epidemic based on the G-Cubed (Asia Pacific) model, which indicated that the economic damage caused by the SARS epidemic on the Chinese mainland that year was estimated to be 1.05% of GDP. Smith [10] also pointed out that although the SARS epidemic was not large-scale, it had a serious and disastrous impact on the economy. Yang et al. [6] examined the impact of the SARS epidemic in 2003 on the Chinese economic system and found that the SARS epidemic had a negative impact on consumption, production price index and transportation, increasing consumer prices and budgetary expenditures. Zheng et al. [11] specifically compared the sales changes of sub-categories of the consumer industry before and after the outbreak of SARS, and found that the sales of food and other daily necessities maintained a steady growth rate, while the sales of clothing, sports and entertainment, furniture and automobiles declined. However, sales growth of pharmaceuticals and home appliances bucked the trend and rose.

After the outbreak of the COVID-19 epidemic, many researchers have generally paid attention to the impact of the COVID-19 epidemic on industrial sector, and believe that the impact of major public health emergencies on the economic system is gradually spread and enlarged through the conduction between industry departments, which leads to an increase in overall economic risks [5, 6, 12, 13]. And most of the literature in this area has examined the changes in the stock market caused by the impact of the epidemic. Yang et al. [5] used the stock market data to analyze the impact of COVID-19 impact on the spillover effect of the industry sector in 2020, and found that the risk spillover effect of various departments after COVID-19 was significantly enhanced. Specifically, the risk of financial, real estate, information technology and consumer departments has increased significantly, while medical, public undertaking and manufacturing departments are risk bearers. Yan and Qian [14] used an event study to examine the impact of COVID-19 epidemic on Chinese consumer sector stock prices and found that consumer sector stock prices fell sharply after the outbreak, but quickly recovered. This indicated that the negative impact was short-lived and transitory. Liu [15] based on Google Trends data from January 1, 2020 to April 12, 2020, using the Generalized Autoregressive Conditional Heteroscedasticity (EGARCH) model, found that the uncertainty caused by the COVID-19 epidemic has caused a significant decline in Chinese stock market index, while leading to greater volatility in stock market indices and industry sector indexes. Shahzad et al. [16] used high frequency data between January 2019 and September 2020 to construct realized upper and lower half variances to examine the impact of the COVID-19 epidemic on the risk spillover effects of Chinese industry sectors using Diebold and Yilmaz model and found that the impact of the COVID-19 epidemic had asymmetric risk spillover effect on various industries in China, and negative volatility spillover dominated. Bouri et al. [17] pointed out that the uncertainty caused by the COVID-19 epidemic had made it easier for global stock market investors to engage in herding behavior, which in turn has led to greater volatility in sector stock prices. Bai and Wei [18] used the Baidu search index combined with the industry stock price data of Chinese listed companies, and used the time-varying parameter vector autoregressive model to examine the relationship between epidemic information and industries, showing that changes in the industrial and consumer industries affect the epidemic information, while changes in epidemic information have a positive output effect on medicine and public utilities. Zeng and Lu [19] on the other hand, used the DCC-GARCH model to analyze the impact of the COVID-19 epidemic on risk spillovers between Chinese stock market and commodity futures markets, and found that the dynamic total spillover effect between stock and commodity markets had increased significantly after the pandemic.

In addition, some other studies had used sector or provincial economic data to assess the impact of COVID-19 epidemic shocks based on input-output relationships across sectors. Liu et al. [13] analyzed the degree of input-output linkage of various industry sectors in Hubei Province based on the perspective of input-output, in order to judge the impact effect and direction of COVID-19. They found that the agricultural, forestry, animal husbandry and fishery products, services, and transportation industries in Hubei Province have strong upstream and downstream influence, and these industries should be given priority protection when implementing epidemic prevention and control measures. Zhu et al. [20] discussed the impact of the impact of COVID-19 on the industrial chain. They believed that the impact of the epidemic caused a capacity gap in my country’s supply chain, which may cause multinational companies to move related industrial chains overseas. Zhang et al. [21] comprehensively used input-output and computable general equilibrium methods to evaluate the impact of COVID-19 on Chinese industries, and pointed out that the comprehensive impact of supply and demand caused by the epidemic will make the construction industry, wholesale and retail industry and real estate industry suffer.

Throughout the research in this area, the existing studies have deepened our understanding of the impact of the COVID-19 epidemic on economic systems and industry sectors from various angles and levels, but deficiencies still exist. On the one hand, the unpredictable and highly contagious nature of COVID-19 poses a great challenge to its prevention and control [22], which also makes the COVID-19 epidemic last for several years. However, the existing literature sample data are mostly until the end of 2020, the sample data collected is too short and the sample size is too small, which is difficult to truly reveal the real evolution process of risk links between industries under the development of the epidemic, and the universality of its research is seriously limited. At the same time, some literatures directly used the SARS epidemic in 2003 as an analogy to estimate the impact of the COVID-19 epidemic shock. Although the SARS epidemic has certain similarities with COVID-19, the duration of SARS is relatively short, and the impact on the social economy is limited, while the duration of COVID-19 lasts for several years, and the impact on the economic system is long-lasting and profound. Therefore, although the conclusions obtained in the earlier literature are of certain reference value, we need to combine samples over a longer period to determine the long-term effects of the COVID-19 shock. On the other hand, although the existing literature has analyzed the economic effects of the COVID-19 epidemic affecting industry sectors from multiple angles and levels. However, most of the existing literature has only measured the degree of industry volatility caused by the COVID-19 epidemic, there are not many relevant literatures on how the impact of the epidemic is transmitted between specific industries. In particular, there is a lack of attention to how the risk linkages between industries fluctuate with the development of the epidemic.

The study in this paper applies daily sample data from a slong period of time before and after the outbreak of COVID-19 from 2016 to 2022, and uses the frontier generalized vector autoregressive model elastic network technology to rolling estimate the connection degree index that can reflect the daily industry risk spillover situation before and after the epidemic. And examines the evolution process of the net spillover effect between industries, comparing the differences in network characteristics between two industries before and after the epidemic, reveals the transmission path of the impact of COVID-19 between industry sectors, and proves the impact of the epidemic on the economic linkages between industries in the medium- and long-term influence. The study finds that the overall risk spillovers of Chinese industries show a dynamic change of "decline-fluctuation-rebound" with the three phases of COVID-19 epidemic. This is a feature not previously found in the empirical research literature based on shorter sample periods. Meanwhile, based on investigating the network characteristics of the two industries, it is found that after the impact of the epidemic, the positive risk spillovers of tourism, hotels, culture, education and sports to other sectors have increased significantly, while the negative spillovers of the financial and real estate industries have increased, and the number of industries affected by information technology and computer industry is significantly lower. This indicates that the risk of the epidemic has been transmitted to the financial and real estate sectors through the tourism, hotel, education and sports industries, thus increasing the overall economic vulnerability. And it shows that there is inter-industry risk transmission of the COVID-19 epidemic shock, and the risk transmission feeds back in a cycle between industries as the epidemic develops, driving the economy into a vicious circle, which was not noticed in the previous literature.

Compared with the literature cited above, the contributions of this paper are as follows. First, this paper uses the sample data of a longer and more updated period, which can fully reveal the evolution of inter-industry risk transmission status under different stages of the development of the COVID-19 epidemic; Second, in response to the characteristics of the vector autoregressive model that requires too many parameters to be estimated, this paper employs a newer elasticity network technique for the estimation of the parameters; Third, this paper is the first to comprehensively and thoroughly examine the impact and transmission mechanisms of epidemic impacts on China’s industry sector networks, which provides the new empirical evidence for academics exploring the links between major public health events and economic risks, and helps to deepen the understanding of academics and policy-making departments on the transmission effects of the industry networks of the COVID-19 epidemic shocks, which has important academic and practical significance.

Next, the structure of this paper is as follows: the second part is the methodology; the third part is findings and discussions; the fourth part is conclusions and insights.

## 2. Methodology

### 2.1. DY model for measuring risk spillover effects

At present, the volatility of financial asset returns is widely used as a risk measurement in the literature, and the volatility correlation between financial asset returns portrays the risk transmission linkages between industries or markets represented by financial assets. The econometric models used to examine risk linkages mainly include the risk spillover model based on vector autoregressive model (VAR) proposed by Diebold and Yilmaz [23–25], and the risk spillover model based on the multivariate GARCH model [26–28], and dynamic conditional correlation model (GARCH-DCC) [29, 30]. Although all of the above models are able to capture volatility spillover effects, but the Diebold and Yilmaz model is relatively more convenient to directly examine the risk output and input relationships among specific industries and has been more widely used in recent years. Therefore, the Diebold and Yilmaz model is used in this paper.

This paper explores the dynamic risk spillover indicators in 20 industrial sectors in China for the period of 2016 to 2022 based on Diebold and Yilmaz [23–25]. According to the idea of Diebold and Yilmaz [23–25], the degree of risk spillover between industries can be obtained by extracting the forecast error decomposition in the vector autoregressive (VAR) model to construct the index of industry connection degree. The industry vector autoregressive model constructed in this paper is as follows:

$$y_{t}=\Psi_{0}+\Psi_{1}y_{t-1}+\Psi_{2}y_{t-2}+\cdots +\Psi_{p}y_{t-p}+\varepsilon_{t}$$ (1)

Where *y*_*t*_ is column vector with N dimensions, composed by N industry stock price volatilities. Ψ_0_ is a matrix of constant items, Ψ_1_, …, Ψ_*p*_ are the coefficient matrices corresponding to the column vectors of the lag phase, *ε*_*t*_ is an independent and identically distributed vector, obeying the N-dimensional normal distribution with the mean vector being 0 and the covariance matrix being Σ. The VAR model (1) can be equivalently described as the following vector moving average distribution form:

$$y_{t}\;=\;{\bar{A}}_{t}\;+\;A_{1}\varepsilon_{t-1}\;+\;A_{2}\varepsilon_{t-2}\;+\cdots +\;A_{t}\varepsilon_{1}\;+\;\varepsilon_{t}$$ (2)

Where ${\bar{A}}_{t}$ is matrix function of Ψ_0_, Ψ_1_, …, Ψ_*p*_. The coefficient matrix *A*_*i*_ of the disturbance term, *i* ≥ 1 follows a recursive expression, see Hamilton [31] for details. Using the standard Cholesky decomposition method for the VAR model, the impulse response based on orthogonal shocks can be obtained, and on this basis, the decomposition components of the forecast error in the future H period can be calculated. However, the standard Cholesky decomposition method requires that the sorting of N economic variables completely conform to the shape of the lower triangle, but this requirement is often difficult to meet in practice. Therefore, following the suggestion of Diebold and Yilmaz [24], we adopt the generalized method of Pesaran and Shin [32] to obtain the prediction error decomposition of the VAR model. In the framework of the generalized VAR model constructed by Pesaran and Shin [32], there is no requirement for orthogonality between N-dimensional shocks, so there is no need to do any orthogonal matrix decomposition, but to use the relationship between the disturbance items caused by a certain shock, and then calculates the generalized forecast error decomposition based on it. Specifically, in the sum of the squares of forecast errors of the volatility of industry i in the future H period, the proportion of the impact from industry j is:

$$\theta_{ij}^{g}(H)\;=\;\frac{\sigma_{jj}^{-1}\sum_{h=0}^{H-1}{\left(e^{\prime }A_{h}\Sigma e_{j}\right)}^{2}}{\sum_{h=0}^{H-1}\left(e^{\prime }A_{h}\Sigma A_{h}^{\prime }e_{i}\right)}$$ (3)

This index actually reflects the degree of connection between industry i and industry j, and the larger the value of this index, the stronger the degree of connection between the two industries. In the generalized prediction error decomposition matrix, the sum of the row vectors is not necessarily equal to 1, and the following standardization can be performed:

$${\bar{\theta }}_{ij}^{g}(H)\;=\;\frac{\theta_{ij}^{g}(H)}{\sum_{j=1}^{N}\theta_{ij}^{g}(H)}$$ (4)

The overall linkage index for all industries can be defined as:

$$S^{g}(H)\;=\frac{\underset{i\neq j}{\sum_{i,j=1}^{N}}{\bar{\theta }}_{ij}^{g}(H)}{\sum_{i,j=1}^{N}{\bar{\theta }}_{ij}^{g}(H)}\times \;100\;=\frac{\underset{i\neq j}{\sum_{i,j=1}^{N}}{\bar{\theta }}_{ij}^{g}(H)}{N}\times \;100$$ (5)

Next, we can define the positive risk spillover effect index of industry i’s impact on all other industries as:

$$S_{.i}^{g}(H)\;=\;\frac{\underset{j\neq i}{\sum_{j=1}^{N}}{\bar{\theta }}_{ji}^{g}(H)}{N}\;\times \;100$$ (6)

Similarly, the negative risk spillover effect index defining industry i affected by all other industry shocks is:

$$S_{i.}^{g}(H)=\frac{\underset{j\neq i}{\sum_{j=1}^{N}}{\bar{\theta }}_{ij}^{g}(H)}{\sum_{i,j=1}^{N}{\bar{\theta }}_{ij}^{g}(H)}\times 100=\frac{\underset{j\neq i}{\sum_{j=1}^{N}}{\bar{\theta }}_{ij}^{g}(H)}{N}\times 100$$ (7)

Based on the above indicators, the net risk spillover effect indicators of the industries of interest in this paper can be calculated, namely:

$$S_{i}^{g}(H)=S_{.i}^{g}(H)-S_{i.}^{g}(H)$$ (8)

In the same way, we can calculate the net risk spillover effect index between two industries:

$$S_{ij}^{g}(H)=\left(\frac{{\bar{\theta }}_{ji}^{g}(H)\;-\;{\bar{\theta }}_{ij}^{g}(H)}{N}\right)\;\times \;100$$ (9)

Compared with the one-way spillover effect index (formulas (6) and (7)), the spillover net effect index can more accurately present the output and input directions of industry risk shocks. Therefore, in the following part of the analysis, we mainly examine the transmission direction of industry risks through the net spillover effect indicators.

### 2.2. Data

This paper uses the daily stock price data of China A-share listed companies from 2016 to 2022 to construct company-level volatility, with a total of 1703 daily samples. The reason why chose to start from 2016 is mainly because of the stock market crash in 2015. During this period, various non-economic fundamental factors interfered, and the stock price rose and fell sharply, which may interfere with the estimation of industry linkages; and from 2016 to 2016. In the period before the outbreak of COVID-19 in 2020, the A-share market was in a relatively stable adjustment stage, without major ups and downs. Meanwhile, in China, the prevention and control of the COVID-19 epidemic began to be relaxed at the end of 2022, and by 2023, the impact of the COVID-19 epidemic on the entire socio-economic life quickly faded, so we chose the sample period until the end of 2022.

According to Diebold and Yilmaz [24], we use the following formula to measure the annualized daily volatility of a single stock i:

$${\tilde{\sigma }}_{it}=100\;\times \;\sqrt{365\;\times \;0.361\;\times \;{\left[ln\left(P_{it}^{max}\right)\;-\;\ln\left(P_{it}^{min}\right)\right]}^{2}}$$ (10)

where $P_{it}^{max}$ is the highest price of stock i on day t, and $P_{it}^{min}$ is the lowest price of stock i on that day. Then we divide the A-share listed companies into 20 industries according to the Wind classification standard, and calculate the annualized daily volatility of the industry weighted by the market value of the market by industry. The specific descriptive statistics of industry volatility are as Table 1.

**Table 1:** Descriptive statistics of industry volatility.

Industry	Energy	Chemicals	Materials	Machinery and Equipment	Enterprise Services	Papermaking and Printing	Transportation Services	Transportation Equipment	Tourism and Hotels	Media and Information Services
Mean	27.5	44.8	43.4	44.3	46.8	41.4	32.9	40.3	43.5	40.8
Median	24.4	41.8	40.8	42.0	43.7	38.0	31.0	37.5	40.4	37.6
Max	106	123	120	127	141	141	110	123	135	126
Min	9.29	23.7	21.2	22.3	19.7	19.2	13.3	17.1	7.39	20.1
Standard Deviation	12.96	13.9	13.7	13.4	15.1	13.7	11.1	14.0	15.3	13.3
Skewness	1.59	1.52	1.50	1.51	1.53	1.97	1.80	1.20	1.47	2.01
Kurtosis	6.66	6.56	6.64	7.28	6.77	9.23	9.26	5.27	6.38	9.33
Industry	Information Technology and Computers	Health Care	Consumer Goods	Medicals	Finance	Real Estate	Culture, Education and Sports	Public Services	Environmental Protection	Agriculture
Mean	46.6	39.6	37.5	40.7	24.6	36.8	47.2	31.2	40.3	43.2
Median	43.8	37.4	35.3	39.1	22.2	33.4	44.6	28.6	36.9	39.2
Max	135	117	102	110	83.0	117	146	102	122	134
Min	21.8	20.0	18.1	18.6	8.82	16.1	18.1	14.3	19.4	15.0
Standard Deviation	14.1	12.1	12.1	13.1	9.91	13.3	16.2	11.6	13.6	16.7
Skewness	1.71	1.92	1.39	1.08	1.62	1.73	1.42	1.85	1.78	1.48
Kurtosis	8.04	9.32	5.88	5.12	6.76	7.66	6.77	8.38	7.86	6.04

It can be seen from Table 1 that there are obvious differences in the volatility distribution of various industries in general. Volatility in energy, finance, transportation services, and public utilities is lower because these industries are basic industries that provide socio-economic necessities and are less sensitive to changes in the economic cycle. The volatility of industries such as chemical industry, materials, machinery and equipment, corporate services, tourism hotels, information technology and computers, medical and health care, culture, education and sports is relatively high, indicating that these industries are highly sensitive to changes in the economic cycle. Under the impact of the new crown epidemic, the degree of risk spillover in these industries is likely to change to a large extent.

## 3. Findings and discussions

### 3.1. Covid-19 and the extent of industry risk spillovers

#### A. Three stages of development of Covid-19

Based on the evolution of the COVID-19, we divide the post-epidemic period into three phases. The first stage starts from January 1, 2020, and ends on December 31, 2020. At this stage, after more than two months of intensive anti-epidemic efforts, the epidemic has basically been eliminated, and only a small number of confirmed cases have reappeared in a few cities. However, the risk of the epidemic has been quickly controlled, and work and production have gradually resumed. The second stage is from January 1, 2021 to February 28, 2022. During this stage, more and more cities across the country have confirmed cases, the number of confirmed cases has increased significantly, and many cities are under lockdown at the same time. The third stage is from March 1, 2022 to December 31, 2022. In this stage, the infectivity of COVID-19 increases, while the fatality rate and severe disease rate decrease. In order to stop the spread of the epidemic, the zero-clearing policy in various places has become increasingly strict, and the production and operation activities of many industries tend to come to a standstill. It was not until December that the epidemic prevention policy became looser.

In the first stage, we expect that industries that have been more affected by the outbreak will show an increase in the net effect of positive spillovers (export risk), that is, the impact of the epidemic will be transmitted to other industries. In the first stage, the industries affected by the impact of the epidemic showed a significant increase in the net effect of negative spillovers (acceptance of external risks). In addition, there are some industries that are less sensitive to the impact of the epidemic, which is manifested in the fact that the fluctuations in the degree of risk spillover in these industries remain basically stable. In the second stage, sectoral industries began to diverge: after adopting strict epidemic prevention measures, some industries gradually returned to normal business activities, and gradually restored foreign economic ties, which showed that the net spillover effect gradually picked up; some industries were strictly cleared Influenced by policies, the vulnerability of the industry has deepened, and it is more susceptible to changes in the external environment. This is manifested in a gradual decline in the net spillover effect, and even a continuous negative net spillover effect. The situation in the third stage is similar to that in the second stage. Except for a small number of industries, the business activities of most industries are affected, and the economic relations between industries fluctuate again. From the above analysis, we can see that with the staged development of the epidemic situation, the degree of risk spillover in specific industries will undergo more complex changes, which cannot be generalized, and only use simple logic to infer. We will analyze it in combination with the specific situation of the industry later.

In order to distinguish the transmission direction of the impact of the epidemic, when presenting the evolution process of the net spillover effect of specific industries, we divide the 20 industries into 4 types of sectors according to the situation in the first stage: the first type is the impact of the epidemic. Industries whose net positive spillover effect has increased significantly; the second type of sector is the impact of the epidemic on the input sector, which is the industry whose net negative spillover effect has increased significantly after the outbreak; the third type is the systemic sector, which maintains a positive net spillover effect before and after the epidemic; the fourth category is vulnerable sectors, that is, industries that maintain a net negative spillover effect before and after the epidemic.

#### B. The impact of the epidemic and overall risk spillover of the industry

We adopt the rolling estimation method to obtain the index value of the industry connection degree of the dynamic risk spillover degree, the rolling estimation window is 200 days, and the lag period of the VAR model is 3 periods. Since there are many parameters in the VAR model, and the sample size in the window period of the rolling estimation is not large, this paper adopts the current common parameter compression estimation when estimating the VAR model. We first give the rolling estimation results of the overall connection degree, see Fig 1 below. To ensure the robustness of the estimated results, we use three parameter compression techniques: Ridge, Lasso, and ElasticNet. Among them, Ridge is a penalty function that adds a quadratic term when estimating parameters, Lasso adds an absolute value penalty function, and elastic network combines the penalty functions of Ridge and Lasso when estimating parameters. It can be seen from Fig 1 that the results obtained by applying the Ridge, Lasso and elastic network methods are basically similar, in which the dynamic trend of the overall connection degree based on the Lasso and elastic network is roughly the same, while the fluctuation range of the overall connection degree index value based on the Ridge method is relatively big. Since the elastic network technique combines the characteristics of Ridge and Lasso, and the estimation results are relatively conservative and robust, only the index values after parameter estimation using the elastic network technology are given in the next part of this paper.

**Fig 1:** The overall risk spillover status of the industry from 2016 to 2022.

The time boundaries of the three phases are marked with red vertical lines in Fig 1. We can see that before the outbreak of COVID-19, the overall connection degree of the industry has remained relatively stable, but after the outbreak of the epidemic, the overall connection degree declined sharply, and then rebounded; but in the second stage, the overall connection degree showed a “decline-recovery” state of repeated fluctuations; in the third stage, the overall degree of connection gradually recovers. It is generally believed that when exposed to a major economic risk shock (e.g., a financial crisis), the degree of linkage across industry sectors should increase (because of the presence of incremental risk output), leading to an increase in overall risk spillovers [25]. Fig 1 shows that after the outbreak of the epidemic, the overall degree of risk spillover among industries has fluctuated greatly, and it has dropped significantly after the outbreak of the epidemic. Taking the index value estimated based on the elastic network as an example, the standard deviation increase of the overall connection degree after the epidemic is about 198% of that before the epidemic, and the maximum decline of the overall connection degree after the epidemic is about 5% of the average connection degree before the epidemic. This reflects the economic system shock characteristics of a major public health event: the epidemic prevention and control policies resulting from a major public health event leads to a reduction in activities and economic linkages across industry sectors, which leads to a decrease in overall industry risk spillovers and fluctuations as the epidemic prevention and control situation evolves. Therefore, the information given in Fig 1 shows that the impact of the epidemic (and the resulting epidemic prevention policy) has changed the original economic relationship between industries. With the change of the epidemic situation (and the resulting change in the epidemic prevention policy), the overall risk spillover also evolved accordingly. However, it is still impossible to know the direction and extent of the impact of the epidemic impact on the risk spread of specific industries from the information on changes in the overall contact degree, and these are the key information we use to judge the transmission path of the epidemic impact. Therefore, next, we will measure the net effect indicators of risk spillovers in 20 industries, and combine them with the changing stages of the epidemic situation to identify the transmission channels of the epidemic impact among specific industries.

#### C. The impact of the epidemic and the evolution of risk spillover of the industry

Fig 2 below shows that industries such as machinery and equipment, papermaking and printing, tourism and hotels, media and information services, and agriculture have seen a significant increase in the net positive spillover effect in the first stage after the outbreak, which means that these five industries have been greatly affected by the epidemic, showing that these five industries are the exporters of the impact of the epidemic and belong to the output sector of the impact of the epidemic. The net spillover effect of the tourism and hotel industry in the first stage reached up to 4.7%, followed by the media and information service industry, with a net spillover effect of up to 3.78%, and the net spillover effect of the paper and printing industry up to 3.2%. It shows that in the first stage, the degree of risk diffusion in tourism hotel industry, media and information industry, and paper printing industry is relatively strong. Judging from common sense, the initial impact (first stage) of the outbreak of the epidemic on the first type of industry has both positive and negative aspects: on the one hand, the epidemic hinders the normal development of the industry’s business activities, leading to a decline in the industry’s prosperity; on the other hand, the epidemic also stimulates demand for products and services related to epidemic prevention. If the impact of the epidemic on a certain industry is mainly negative, when the epidemic continues to develop (the second stage), the industry must be in a relatively depressed state, and the degree of external contact of the industry will inevitably decline, and it is more likely to be affected by other industries (vulnerability revealed). Conversely, if the industry is affected by the increase in demand caused by the epidemic and the prosperity of the industry increases, the impact of this industry on other industries will inevitably expand (systematically manifested). Therefore, based on the changes in the net spillover effect in the first two stages, we can reasonably judge the actual effect of the epidemic on the sector. From Fig 2, it can be seen that in the second stage, the net effect of risk spillovers in this sector declined to varying degrees. Among them, paper printing, media and information services, and agriculture changed from positive effects to negative effects: the net spillover effect of agriculture fell to -4.85%, the paper printing industry fell to -4.39%, and the media and information services industry fell to -3.1%. Although the machinery and equipment and tourism and hotel industries still maintain a positive net spillover effect, the degree of risk correlation has dropped significantly during this period: the net spillover effect of the machinery and equipment industry has dropped from the highest 4.44% to -1.3%, and the tourism and hotel industry has dropped to -1.3%. These circumstances show that the impact of the epidemic has a negative impact on the sector. In the third stage, the net spillover effect of the machinery and equipment industry, paper printing, and media and information service industries fluctuated significantly, while tourism, hotels and agriculture were more negatively affected by the epidemic, and continued to maintain a negative net spillover effect.

**Fig 2:** The evolution of industry risk spillovers in the output sector impacted by the epidemic.

Fig 3 below shows that industries such as materials, transportation equipment, commercial trade, medical and health care, and environmental protection have obvious negative spillover net effects in the first stage after the outbreak, which means that these five industries have been affected by other industries after the outbreak. The greater impact of the industry shows that these industries are the recipients of the impact of the epidemic and belong to the input sector of the impact of the epidemic. Among them, the industry with the largest negative net spillover effect is the environmental protection industry, which reached -4.32% at this stage; the second is the commercial trade industry, which reached -3.37%; the third is the transportation equipment industry, which reached -2.82%. We can see that after the three industries of transportation equipment, commercial trade and medical and health experienced the first stage of external shocks, the second stage began to have a net positive spillover effect, suggesting that these three industries will gradually resume normal business activities in the second stage. At the same time, due to the increase in demand caused by the epidemic, the industry is showing a structural boom. But in the third stage, affected by the increasingly stringent epidemic prevention and control policies, the commercial trade and medical and health industries have endured more impacts from external industries. The materials industry belongs to the upstream industry, suffering the impact of external demand from the middle and downstream industries in the first and second stages after the outbreak of the epidemic, and gradually adjusting in the third stage. During the epidemic, as the demand for environmental protection services and products in the external industry continued to weaken, the environmental protection industry has been affected by the impact of negative external demand, resulting in an increasing net negative spillover effect.

**Fig 3:** The evolution of industry risk spillovers in the input sector impacted by the epidemic.

Figs 4 and 5 below respectively show the evolution of industry risk spillovers in the systemic sector that continues to export risks externally and the vulnerability sector that continues to receive external risks. The industries that belong to the systemic sector are chemical industry, enterprise services, information technology and computer, culture, education and sports, and the industries that belong to the vulnerable sector are energy, transportation services, consumer goods, finance, real estate and public utilities. Combining the information in Figs 4 and 5, we can find that although the direction of the spillover effects of the two sector industries is basically the same before and after the epidemic, the fluctuations of the spillover effects of the two sector industries after the epidemic are greater than before the epidemic. Meanwhile, it should be noted that the influence of the information technology and computer industry on other industries continued to rise before the epidemic, but after the outbreak, although the positive external impact was maintained, the degree of influence was weakening day by day. The net spillover effect slipped from 6.42% at the peak of the first phase to 0.3% at the lowest of the second phase, and has since recovered. These results imply that the informatization process of other industries has been hindered to a greater extent during the epidemic prevention and control period, which may affect the future growth potential of other industries. In addition, the culture, education and sports industry has maintained a relatively high net positive spillover effect during the epidemic, indicating that the culture, education and sports industry is playing an increasingly important role in my country’s economic system, and its role in driving other economic sectors is becoming more and more important.

**Fig 4:** Evolution of industry risk spillovers in systemic sectors.

**Fig 5:** Evolution of industry risk spillovers in vulnerable sectors.

Overall, from the analysis of the three stages of the net risk spillover effects for each industry sector, we can see that the industries in which positive risk spillover effects occurred at the beginning of the outbreak reversed their risk spillover effects when the outbreak progressed to the second or third stage: the positive effects declined or even the net risk spillover effects became negative. This indicates that there is a negative feedback loop in the risk transmission, and the epidemic shock keeps spreading through the negative feedback loop, which may lead to a vicious circle in the overall economy. Therefore, in order to avoid the expansion of the negative impact caused by the epidemic shock, policy departments should keep abreast of the dynamic changes of the risk output and input of the epidemic shock and take strong measures to block the risk transmission of the epidemic for specific industry sectors.

### 3.2. Comparison of industry network characteristics

The previous session discussed the evolution of risk spillovers in various industries before and after the outbreak of COVID-19. Although it helps us to find out the transmission process of the impact of the epidemic, we still do not know much about the specific inter-industry economic risk linkages. In this section, we will further examine the changes in network relationships between industries before and after the epidemic, in order to better understand the impact of COVID-19 on industry risk linkages. We divide the samples into pre-COVID-19 (January 1, 2016 to December 31, 2019) and post-epidemic (January 1, 2020 to December 31, 2022), and then according to formula (9) we estimate the net spillover effect indicators between two industries respectively, selecting the industry samples belonging to the highest 10% of the spillover effect to construct the industry association network. Based on this, the industry network diagram before and after the epidemic is shown in Fig 6 below.

**Fig 6:** Industry connection before the epidemic.

Comparing Figs 6 and 7, we can find that there have been significant changes in industry network relationships before and after the impact of the epidemic: the economic risk linkages of some industries have increased, but those of other industries have decreased; after the epidemic, the direction of risk spillovers in some industries has even reversed. Before the epidemic, there were very few industrial network connections important to the tourism and hotel industry, which was mainly affected by the information technology and computer industry, and also affected the energy industry including water, electricity and heating. After the epidemic, the network connection of this industry has increased significantly, which has a large positive spillover effect on industries such as consumer goods, finance, energy, and agriculture, and has become the exporter of epidemic risks. This is mainly due to the outbreak of the COVID-19 epidemic, which has caused a more pronounced and direct impact on the tourism and hotel industry (from a sharp decline in tourism numbers and a significant drop in industry performance) and the demand for related goods, services and services in the tourism and hotel industry has declined, which in turn has affected the consumer goods, finance, energy, agriculture and other industries, deepening the external impact on these industries. Before the epidemic, the culture, education and sports industry were mainly affected by the information technology and computer industry, and had no other important industry connections. After the outbreak of the epidemic, the business activities of the culture, education and sports industry were affected by the epidemic prevention and control, and it had significant positive spillover effects on consumer goods, finance, energy, environmental protection and agriculture through the demand channel. The financial industry and the real estate industry have been significantly impacted by other industries after the epidemic, indicating that these two industries have become more vulnerable after the epidemic. The information technology and computer industry had an important impact on 9 industries before the epidemic, but only 4 industries after the outbreak, implying that the outbreak of the epidemic has seriously hindered the popularization and promotion of information technology and intelligent technology, which deserves attention. The environmental protection industry had a relatively important impact on the five industries before the epidemic, reflecting the implementation of the national environmental protection policy; but after the outbreak of the epidemic, the influence of the environmental protection industry on other industries has declined. On the contrary, changes in other industries have affected the environmental protection industry.

**Fig 7:** Industry connection after the outbreak.

## 4. Conclusion

Large-scale infectious disease outbreaks have always been public health emergencies that seriously threaten human health and social security, and have a serious impact on the economic operation system. COVID-19 lasted a long time, and the wide range of faces was rare since the founding of the People’s Republic of China, and it has had a long-lasting and profound impact on the Chinese economy. The existing literature still lacks research on the risk transmission pathways of the COVID-19 epidemic impact and the changes in the characteristics of industry contact networks caused by the epidemic. This paper applies ElasticNet method proposed by Diebold and Yilmaz [23–25] to estimate the dynamic risk spillover indicators of 20 industry sectors in China from 2016 to 2022, and systematically examines the impact of industry risk network fluctuations and the transmission path caused by COVID-19 shock. The results of this study are as follows:

1. The impact of COVID-19 epidemic has caused a large fluctuation in the overall risk spillover of Chinese industry. The standard deviation of the overall linkage increased by about 198% of the pre-epidemic level, and the maximum decrease of the overall linkage after the epidemic was about 5% of the average linkage before the epidemic. With the three phases of the COVID-19 epidemic, the overall risk spillovers of Chinese industries show a dynamic change of "decline-fluctuation-rebound", which is a feature not found in the previous empirical research literature based on a shorter sample period, and reflects the difference between the impact of major public health event shocks and general economic risk shocks on the economic system.
2. As the epidemic develops, the risk spillover of various industries has shown dynamic characteristics of mutual influence. At the beginning of the epidemic, machinery and equipment, paper and printing, tourism and hospitality, media and information services, and agriculture were the net exporters of epidemic risks, while materials, transportation equipment, commercial trade, medical and health care, and environmental protection were the importers of epidemic risks. However, the risk spillover from these sectors reverses to some extent in the subsequent period, and these circumstances imply that the risk exporting sectors at the beginning of the epidemic are likely to be subject to negative feedback shocks from other sectors in the subsequent period.
3. Based on investigating the network characteristics of the two industries, it is found that after the impact of the epidemic, the positive risk spillovers of tourism, hotels, culture, education and sports to other sectors have increased significantly, while the negative spillovers of the financial and real estate industries have increased, and the number of industries affected by information technology and computer industry is significantly lower. This indicates that the risk of the epidemic has been transmitted to the financial and real estate sectors through the tourism, hotel, education and sports industries, thus increasing the overall economic vulnerability. It is worth noting that the spillover effect of information technology and computer industry to other industries declined significantly during the epidemic, indicating that the epidemic hindered the promotion of information technology, which was not noticed in the previous literature.

The contribution of this study lies in using the newer and longer sample data, the use of more cutting-edge elastic network technology, the discussion of the output and input side of industry risks under the impact of the new crown epidemic, and the in-depth investigation of the changes of industry risk spillover in the three stages of epidemic development and the changes of industry network characteristics, and obtained many new findings and conclusions.

The contribution of this study is that it explores the output side and input side of industry risk under the impact of the COVID-19 epidemic by using updated and longer period sample data and employing the more cutting-edge elastic network technique, and it also makes an in-depth examination of the changes of industry risk spillover and network characteristics in the three stages of epidemic development, and obtains a number of new findings and conclusions. This paper shows that due to the interdependence between sectors of the economic system, the transmission direction and transmission effect of epidemic risk between industry sectors are not fixed, and the risk exporting industry is likely to be affected by the risk input industry in the subsequent period, which leads to a vicious circle in the economic system. How to block the occurrence of this vicious cycle depends on our in-depth understanding of the dynamic evolutionary paths and transmission mechanisms of the economic system impacted by the COVID-19 epidemic. It is particularly noteworthy that this paper finds that the service sector was the main export sector of the epidemic risk during the epidemic, the application of information technology has been hindered, the financial and real estate sectors have been affected by external shocks, and the overall economic vulnerability has increased. Therefore, relevant departments should pay attention to and play the role of the service sector in blocking the spread of negative shocks of the epidemic, pay close attention to the risks of the financial and real estate sectors to avoid black swan events, and increase support for IT applications to hedge against the negative impacts of the epidemic. Of course, the research in this paper still has certain limitations, due to the large differences in the models and sample data used to examine the various literature on the impact of the new crown epidemic, it is still difficult to make a more accurate quantitative comparison of the differences in risk spillover effects in different literature. In the future study, we intend to examine the effects of empirical tests of multiple quantitative models of risk spillover over a longer sample period simultaneously to gain a more comprehensive understanding of the risk transmission mechanism under the COVID-19 epidemic shock.

## Supporting information

S1 Data (ZIP)
